This article has been retracted.

# Gut microbiota and COVID‐19: A systematic review

**DOI:** 10.1002/hsr2.1080

**Published:** 2023-01-27

**Authors:** SeyedAhmad SeyedAlinaghi, Arian Afzalian, Zahra Pashaei, Sanaz Varshochi, Amirali Karimi, Hengameh Mojdeganlou, Paniz Mojdeganlou, Armin Razi, Farzaneh Ghanadinezhad, Alireza Shojaei, Ava Amiri, Mohsen Dashti, Afsaneh Ghasemzadeh, Omid Dadras, Esmaeil Mehraeen, Amir Masoud Afsahi

**Affiliations:** ^1^ Iranian Research Center for HIV/AIDS, Iranian Institute for Reduction of High Risk Behaviors Tehran University of Medical Sciences Tehran Iran; ^2^ School of Medicine Tehran University of Medical Sciences Tehran Iran; ^3^ Department of Pathology Urmia University of Medical Sciences Urmia Iran; ^4^ Shahid Beheshti University of Medical Sciences Tehran Iran; ^5^ Shahid Chamran University of Ahvaz Ahvaz Iran; ^6^ Department of Radiology Tabriz University of Medical Sciences Tabriz Iran; ^7^ Department of Global Public Health and Primary Care University of Bergen Bergen Norway; ^8^ Department of Health Information Technology Khalkhal University of Medical Sciences Khalkhal Iran; ^9^ Department of Radiology University of California, San Diego (UCSD) California USA

**Keywords:** COVID‐19, gut microbiota, microbiome, microbiota, probiotics, SARS‐CoV‐2

## Abstract

**Background and Aims:**

Alteration in humans' gut microbiota was reported in patients infected with severe acute respiratory syndrome coronavirus‐2 (SARS‐CoV‐2). The gut and upper respiratory tract (URT) microbiota harbor a dynamic and complex population of microorganisms and have strong interaction with host immune system homeostasis. However, our knowledge about microbiota and its association with SARS‐CoV‐2 is still limited. We aimed to systematically review the effects of gut microbiota on the SARS‐CoV‐2 infection and its severity and the impact that SARS‐CoV‐2 could have on the gut microbiota.

**Methods:**

We searched the keywords in the online databases of Web of Science, Scopus, PubMed, and Cochrane on December 31, 2021. After duplicate removal, we performed the screening process in two stages; title/abstract and then full‐text screening. The data of the eligible studies were extracted into a pre‐designed word table. This study adhered to the PRISMA checklist and Newcastle−Ottawa Scale Bias Assessment tool.

**Results:**

Sixty‐three publications were included in this review. Our study shows that among COVID‐19 patients, particularly moderate to severe cases, the gut and lung microbiota was different compared to healthy individuals. In addition, the severity, and viral load of COVID‐19 disease would probably also be influenced by the gut, and lung microbiota's composition.

**Conclusion:**

Our study concludes that there was a significant difference in the composition of the URT, and gut microbiota in COVID‐19 patients compared to the general healthy individuals, with an increase in opportunistic pathogens. Further, research is needed to investigate the probable bidirectional association of COVID‐19 and human microbiome.

## 1 INTRODUCTION

At the early ages of human life, diverse viruses, bacteria, and fungi colonize the skin, oral cavity, and gut. These microorganisms are known as the “human microbiota”^1^, ^2^ The various microorganisms that colonize the gastrointestinal (GI) tract in a complex and dynamic ecosystem are termed the “gut microbiota.”^3^, ^4^ The number of microorganisms inhabiting the GI tract is estimated to surpass 10^14^, which have ten times more bacterial cells than the number of human cells and about 150 times more genes (microbiome) than the human genome.^3^, ^5^

The eubiosis is defined as an interspecies balance of the microbiota community that is dominated by members of mostly these four bacterial phyla, including^1^ Actinobacteria,^2^ Bacteroidetes,^3^ Firmicutes, and^4^ Proteobacteria. Any change in gut bacterial composition or disruptions in the hemostasis of gut microbiota is called “dysbiosis.”^6^ During human life, gut microbiota provide numerous benefits, such as food digestion, crucial vitamins production, biliary acids deconjugation, and other essential biochemical benefits.^4^, ^7^ The gut microbiota also interacts with the immune system by controlling the pathogens load with direct competition for limited nutrients, and has recently been shown to have a regulatory relationship with organs such as the lung, known as the “gut‐lung axis.”^8^, ^9^ For instance, more than 50% of patients with inflammatory bowel disease (IBD) and 33% of patients with irritable bowel syndrome are prone to respiratory disorders due to dysbiosis without a history of chronic or acute respiratory disease.^10^, ^11^

The novel corona virus which triggered severe acute respiratory syndrome coronavirus‐2 (SARS‐CoV‐2),^12^, ^13^ also showed to have effects on GI and upper respiratory tract (URT) microbiota and frequent symptoms were anorexia, diarrhea, nausea/vomiting, and abdominal pain.^14^, ^15^, ^16^ Few studies discovered dysbiosis and a rise in GI opportunistic microorganisms in patients infected with SARS‐CoV‐2 that suggested a possible link between the gut‐lung axis and SARS‐CoV‐2.^17^, ^18^

The human URT is the main entrance for aerosol transmission of infection, including SARS‐CoV‐2, and is a notable reservoir of SARS‐CoV‐2.^19^, ^20^ The most frequent microbiotas in the oral and URT are the Streptococcus spp.^21^ COVID‐19 also has a notable effect on lung microbiota, especially with potential dysbiosis and a rise in opportunistic microorganisms in URT.^22^, ^23^

An obvious association exists between the overall health of the gut microbiome and the progression of COVID‐19. Additionally, the altered gut microbiota has been shown to persist in patients even after several days up to 6 months after clearance of COVID‐19.^24^, ^25^ Also, poor outcome were reported in elderly or comorbid patients.^26^, ^27^ Recently, several studies discussed the factors associated with the dysbiosis in COVID‐19 patients manifesting GI symptoms. According to some research, increased inflammation may lead to a “leaky gut,” which permit the transfer of bacterial metabolites and toxins into the systemic circulation.^27^ This might cause further complications to the severe COVID‐19 patients.^24^ Besides, interventions targeting to re‐establish a correct microbiota composition are important for developing a more comprehensive approach to managing COVID‐19.^28^

Therefore, reviews and critical assessments of the rapidly developing research evidence on this significantly important issue are extremely necessary. Accordingly, we aimed to systematically review the effects of gut microbiota on the SARS‐CoV‐2 infection and its severity and also the impact that SARS‐CoV‐2 could have on the gut microbiota.

## 2 METHODS

To ensure the goals, this study adheres to the Preferred Reporting Items for Systematic Reviews and Meta‐Analyses (PRISMA) checklist.

### 2.1 Data sources

We first found the related keywords using the previously published studies and the medical subject heading (MeSH) database. After designing a search strategy, we searched the keywords in the databases of Web of Science, Scopus, PubMed, and Cochrane on December 31, 2021. Supporting Information Material 1 contains the search strategies for all the databases. The search terms for PubMed areas below:

1. “Novel coronavirus” or “2019‐nCoV” or “SARS‐CoV‐2” or “COVID‐19” or “SARS‐CoV2” [Title/Abstract]
2. “Gut microbiota” or “Microbiota” or “Gastrointestinal microbiome” or “Microbiome” or “Microflora” or “Probiotics” or “Prebiotics” or “Microbial Community” [Title/Abstract]
3. [A] AND [B].

### 2.2 Study selection

The eligible studies were selected in two steps. First, four researchers screened and selected the studies based on the relevancy of titles and abstracts. In the second step, the same group of researchers went through the full texts of the remaining studies and selects the most relevant studies against the eligibility criteria of the present study. Any disagreements between the researchers were addressed by another independent researcher to resolve the inconsistencies in the results.

The original studies that evaluated the relationship between gut microbiota and COVID‐19 (either the effect of microbiota on the COVID‐19 or the effect of SARS‐CoV‐2 on microbiota) were considered eligible.

The exclusion criteria were as follows:

1. Abstracts, conference abstracts, or studies without published full text.
2. Non‐original studies, including opinions and review articles.
3. Case reports.
4. Nonhuman studies.

### 2.3 Data extraction

Four researchers went through the full texts of the selected documents in the final stage and extracted the necessary information for included studies such as the first author name, country of study, year of publication, type of studies, the population mean age, sampling location, type of microbiota, how microbiota affect the course of COVID‐19 disease and vice versa, how SARS‐CoV‐2 infection affects the microbiota, and summary of other findings. Table 1 shows the summary of extracted data. Other team members double‐checked the results and selected records to refrain from any probable remaining duplications and/or overlaps.

### 2.4 Quality and bias risk assessment

As above‐stated to ensure the authenticity and reliability of the outcomes, this study abides by guidelines of the PRISMA protocol. Additionally with the purpose of minimizing Bias Risk we have utilized Newcastle−Ottawa Scale (NOS) to evaluate the studies. This scale consists of three items of selection, comparability, and exposure/outcome. These items are graded maximum scores of 4, 2, and 3 respectively. Maximum score of 9 is allocated for individual studies by adding up these values (Table 2).

**Table 1:** Summary of findings for the included studies.

ID	First author	Countries	Year of publication	Type of study	Population (no, mean age ± SD)	Sampling location	Type of microbiota	How microbiota affect the course of the COVID‐19	How SARS‐CoV‐2 infection affect the microbiota	Summary of findings
1	^40^	UAE	2021	Cross‐Sectional	*N* = 143	Fecal	Intentinibacter Enterorhabdus Anaerostipes Prevotella Bacteroides Bifidobacterium Blautia Faecalibacterium Streptococcus Lachnospiraceae Atopobiaceae Peptostreptococcaceae	No relation between COVID‐19 viral load and bacterial microbiome Decreases severity of COVID‐19 disease	Gut microbiota diversity↑. Blautia↑ Faecalibacterium↑ Streptococcus↑ Intestinibacter↓ Enterorhabdus↓ Anaerostipes↓ Bifidobacterium↓ Bacteroides↓ Prevotella↓	Stool in COVID‐19 infected patients: richer, more variable in bacteria specie+ high lipid metabolism Gut microbiota is protective against severe COVID‐19 disease.
2	^45^	Saudi Arabia	2020	Experimental	‐	‐	Lactobacillus plantarum probiotics bacteria	Lactobacillus plantarum metabolites (Plantaricin BN, Plantaricin JLA‐9, Plantaricin W, Plantaricin D) can bind with RdRp, RBD, and ACE2 molecules.	‐	Plantaricin molecules can be useful against the COVID‐19 disease.
3	^41^	Hungary	2021	Cross‐sectional	*N* = 40 Age Athlete (*n* = 20): Age = 24.15 ± 4.7 years, Sedentary (*n* = 20): Age = 27.75 ± 7.5	Fecal	Actinobacteria Bacteroidetes Cyanobacteria Firmicutes Proteobacteria Tenericutes Verrucomicrobia	Decreases symptoms of Severe COVID Bacteroidetes↑	Bacteroidetes↑	Bacteroidetes in the feces have an anti‐inflammation effect and protect patients against severe COVID‐19 disease. No difference between the microbiome of athletes and sedentary patients
4	^70^	Iran	2021	Basic	‐	‐	Lactobacillus Plantarum Bos taurus Bacillus subtilis Morone saxatilis Crotalus durissusruruima Leuconostocgelidum Lachesanatarabaevi Limulus polyphemus	glycocin F (from Lactococcus lactis) and lactococcine G (from Lactobacillus Plantarum) have the highest affinity to some SARS‐COV‐2 virus molecules.	‐	Using dairy products containing Lactococcus lactis and Lactobacillus Plantarum with vitamin D may be helpful to combat and preventing SARS‐COV‐2 infection.
5	^76^	Turkey	2021	Cross‐sectional	*N* = 44	‐	Bifidobacterium	Single strain probiotic bifidobacterial: mortality rate↓ duration of admission ↓ (in moderate/severe COVID‐19 patients) This probiotic also helps chest CT‐Scan resolution.	‐	Bifidobacterium can be a useful treatment for moderate/severe COVID‐19 disease.
6	^42^	China	2021	Cross‐sectional	*N* = 28703 (1374 CRC patients) + 27,329 normal patients	Colon	Melissococcus, Faecalibacterium, Subdoligranulum, Bacteroides, Alistipes, Eubacterium, Parabacteroides, Ruminococcus, Blautia, Bifidobacterium.	Blautia and Ruminococcus are more prevalent in CRC (colorectal cancer) patients and are related to a more severe COVID‐19 disease in these patients.	‐	The imbalance of gut microbiota is related to COVID‐19 mortality.
7	^66^	China	2021	Prospective Study	*N* = 30 median age: 53.5	Gut		The imbalance of gut microbiota is linked to long COVID. Higher CRP levels in patients with reduced postconvalescence microbiota richness.	Gut microbiota changes in the COVID‐19 patients. microbiota richness did not normalize after a 6‐month recovery	Enhancing the microbial diversity of the gut in long COVID‐19 patients should be considered. Severe patients had lower postconvalescence microbiota richness.
8	^43^	Germany	2021	Cross‐Sectional	*N* = 322 Healthy (*n* = 72, Median age=36) URT (*n* = 112, Median age = 46) Mild COVID (*n* = 36, Median Age = 50) Moderate COVID(*n* = 37, Median Age = 57) Severe COVID (*n* = 65, Age = 65)	Oropharyngeal	Haemophilusin fluenzeae Parainfluenzae pittmaniae Neisseria subflava		↓nasopharyngeal microbiota diversity (in admitted COVID‐19 patients) Microbiota of moderate/severe COVID‐19 patients was more dysbiotic than in healthy patients. Haemophilus influenzeae↑ parainfluenzae↑ pittmaniae↑	Gut microbiota changes: Moderate and severe COVID‐19 patients Patients treated with antibiotics. History of mechanical ventilation during the admission. Prolonged hospitalization.
9	^44^	Italy	2021	Cross‐Sectional	49 Mean Age = 66.7 ± 14.4	Gut	Actinobacteria Bacteroidetes Firmicutes Proteobacteria Verrucomicrobia		Bacteroidetes was seen more in COVID + patients and decreased after recovery. Firmicutes were seen in COVID‐ patients (and after recovery of COVID+ patients). Blautia ↑ (after recovery)	Alpha diversity: similar in COVID+ and COVID− pneumonia alpha‐diversity ↑ (after the recovery)
10	^20^	Italy	2021	Cross‐Sectional	*N* = 40	Nasopharynx	Actinobacteria Bacteroidetes Firmicutes Fusobacteria Proteobacteria		Bacterial richness, diversity, and abundance were similar in both COVID+ and COVID− groups (mild disease)	Nasopharyngeal microbiota does not change in mild early COVID‐19 disease.
11	^48^	USA	2021	Experimental	~78 Samples	Lung and blood microbiome	(Long list)	blood microbiota COVID‐19 patients: E. coli, Bacillus sp. PL‐12 abundance, Campylobacter hominis ATCC BAA‐381 Pseudomonas sp. I‐09 Thermoanaerobacter pseudethanolicus ATCC 33223 Thermoanaerobacter iumthermosaccharolyticum DSM 571 Staphylococcus epidermis Less severe SARS‐CoV‐2 infection with Bacillus subtilis subsp. subtilis str. 168 blood	Multiple associations were seen between microbiota and COVID‐19 severity.	Interleukins modulation by the microbiota (lung and blood) results in immune system regulation.
12	^46^	USA	2021	Cross‐Sectional	*N* = 19 (9 COVID positive: Mean ± (SD) = 53.38 ± (14.93)) 10 COVID negative.	nasopharyngeal	Proteobacteria, Actinobacteria Firmicutes, Corynebacterium, Morganella Moraxella, Escherichia‐Shigella, Proteus Staphylococcus	‐	Alpha‐diversity analysis:same in COVID+ and COVID− beta‐diversity: significant variation richness ↓ in COVID+ Proteobacteria‐to Actinobacteria ratio↑in COVID+	In COVID + patients: Dysbiotic nasopharyngeal microbiota Loss of normal flora bacteria. pro‐inflammatory bacteria. ↑
13	^47^	USA	2021	Cohort	118 IBD patients	Gut (Endoscopy)	‐	‐	No change in the endoscopic microbiome of 12 IBD before and after SARS‐CoV‐2 infection was seen	No change in microbiota.
14	^50^	Italy	2021	Cross‐Sectional	*N* = 69 Mean Age = 73 years	Fecal	Enterococcaceae, CoriobacteriaceaeLactobacillaceae, Veillonellaceae, PorphyromonadaceaeStaphylococcaceaeBacteroidaceae, LachnospiraceaeRuminococcaceaePrevotellaceaeClostridiaceae	‐	High Dysbiosis of gut microbiota in COVID+ patients. ↓(Alpha)diversity, ↓Firmicutes, Bacteroidetes, ↑Enterococcaceae, Coriobacteriaceae,	In COVID patients: Loss of beneficial microorganisms ↑potential pathogens (ex: Enterococcus especially in ICU patients)
15	^51^	Chili	2020	Cross‐Sectional	>200000	Waste water	(Based on NCBI Taxonomy tree)	‐	↓Proteobacteria and ↑in other genera at the residential care home and the prison during the pandemic. COVID+ samples: ↑Prevotella, Bacteroides, ↑Simpliscira, Flavobacterium, Acinetobacter genera	The microbiota in the waste water of the COVID‐19 patients' region was different compared to the the non‐COVID individuals’ region.
16	^52^	China	2021	Cross‐Sectional	*N* = 400 Mean age: ~47 years	Oropharyngeal	Long list	‐	↓Alpha‐diversity ↑Opportunistic pathogens ↓butyrate‐producing genera In COVID+: ↑Firmicutes. ↑Bacteria_unclassified	↑The beta diversity Dysbiosis + (In COVID+) COVID‐19 patients: lipopolysaccharide‐producing bacteria ↑Leptotrichia ↑opportunistic pathogens (Granulicatella) ↓Butyrate‐producing bacterial
17	^53^	India	2021	Cross‐Sectional	*N* = 89	nasopharyngeal	OUT (Long list)		COVID+: ↓Number of Bacteria ↑Proteobacteria ↓Bacteroidetes ↑opportunistic pathogens (Haemophilus, Stenotrophomonas, Acinetobacter, Pseudomonas): ↑Chance of secondary infection. ↔Bacterial richness	In mild cases of COVID‐19 dysbiosis level returns to normal values in a short time after the recovery. In children normalization takes more time.
18	^55^	USA	2021	Cross‐Sectional	164 Mean age: ~63 years	Oral		Long COVID patients had inflammatory microbiota (ex. Prevotella, Veillonella which produce LPS):		Long COVID and chronic fatigue syndrome patients had similar oral microbiome. Malfunction of oral microbiota is associated with long COVID symptoms. Decreased anti‐inflammatory metabolic pathway was seen in oral microbiota of long COVID patients
19	^57^		2021	Cross‐Sectional	*N* = 7	Fecal		‐	↓Actinobacteria, ↓Firmicutes, ↓↓Bacteroidetes	↓Shannon Diversity Index (In COVID+)
20	^77^	Egypt	2021	Cohort	*N* = 200 Mean age = 37 (Mild COVID‐19), 45 (moderate COVID‐19)	‐	‐	Prebiotic‐containing foods, low sugar diet, exercise, adequate sleep, and less antibiotic use cause a milder COVID‐19 disease. Intake of probiotic yogurt :1.6 times greater risk of severe COVID‐19 disease.	‐	A healthy gut microbiome can decrease the severity of COVID‐19. But probiotic yogurt may be harmful and has an adverse effect on COVID progression.
21	^31^	Mexico	2021	Cross‐Sectional	*N* = 95 Mean age: 45 years	Upper respiratory tract	Most Common: Firmicutes, Bacteroidetes, Proteobacteria	Loss of microbial complexity structure changes prognosis of SARS‐CoV‐2 infection	↑Firmicutes, ↑Actinobacteria, ↑TM7 ↑Veillonella, ↑Staphylococcus, ↑Corynebacterium, ↑Neisseria, (Only in severe SARS‐CoV‐2 infection) ↓Bacteroidetes ↓Haemophilus ↓Alloiococcus	High dysbiosis in the respiratory microbiome of COVID‐19 patients ↓microbial diversity ↑Firmicutes/Bacteroidetes mild COVID: ↑Prevotellamelaninogenica, P. pallens, Veillonella parvula, Neisseria subflava, In Severe COVID: ↑Megasphaera, CW040. Fatal COVID: ↑ Rothiadentocariosa, Streptococcus infantis, Veillonelladispar
22	^58^	Bangladesh	2021	Cross‐sectional	*N* = 22 mean age: 41.86	Nasopharyngeal	2281 bacterial species		Opportunistic bacteria 67% of acute SARS‐CoV‐2 infection cases. (in 77% of recovered patients) In acute and recovered COVID‐19 patients 79% of healthy common bacteria were not detected in. alpha‐diversity: higher diversity in Recovered > Healthy > Acute COVID	Nasopharyngeal microbiome dysbiosis in SARS‐CoV‐2 infection decreases the diversity of the nasopharyngeal microbiome and can change the genomic of microbiomes.
23	^59^	USA	2021	Prospective cohort	*N* = 274 Children. Median Age: Healthy: 9.2 Infected (without respiratory symptoms): 9.1 Infected + respiratory symptoms: 14.2	Nasopharyngeal	1799 ASVs 316 bacterial genera 20 phyla		(Nasopharyngeal microbiome alpha diversity: no difference. Microbiome richness ↑ in COVID+ In respiratory involved SARS‐CoV‐2 infection: ↑Corynebacterium, ↑Anaerococcus spp.	High Corynebacterium in the nasopharyngeal microbiome In SARS‐CoV‐2 infection. ↑Dolosigranulumpigrum in nasopharyngeal tissue is associated with SARS‐CoV‐2 infection (Not respiratory involvement). COVID‐19 can change the nasopharyngeal microbiome composition in children.
24	^60^	Italy	2021	Pilot study	*N* = 41 Mean Age: 47.3	Oral	Haemophilusparainfluenzae, Veillonellainfantium, Soonwooa purpurea, Prevotellasalivae, Prevotellajejuni, Capnocytophagagingivalis Neisseria perflava,		↓Richness (↓alpha diversity) Difference in beta‐diversity: ↑Prevotellasalivae ↑Veillonellainfantium Healthy: ↑Neisseria perflava ↑Rothiamucilaginosa	Different microbiota composition was seen in COVID+ patients. Seven cytokines in the oral microbiome of the COVID patients: IL‐6, IL‐5, GCSF, IL‐2, TNF‐a, GMCSF, INF‐γ
25	^29^	Russia	2021	RCT	*N* = 200, Mean age = 65 (59–71) [probiotic group] 64 (54–70) [nonprobiotic groups]		The probiotic receiving group was treated with; rhamnosus PDV 1705, Bifidobacterium bifidum PDV 0903, Bifidobacterium longum subsp. infantis PDV 1911, and Bifidobacterium longum subsp. longum PDV 2301 for 14 days.	In COVID‐19 patients, the tried probiotic had no noteworthy impact on the severity of the disease or mortality.		In this study, the tried probiotic was beneficial to treat diarrhea in COVID‐19 patients.
26	^30^	China	2020	Observational	*N* = 800			Probiotics were helpful to treat COVID‐19 diarrhea.		
27	^61^	Korea	2021	Cross‐Sectional	*N* = 48 Median age: 26 year	Fecal	16 S rRNA amplicon sequencing		In respiratory COVID+ **Firmicutes** > Proteobacteria > Actinobacteria> Bacteroidetes ↓Bacteroidetes,	The microbial diversity of COVID infected was higher than recovered cases. acute SARS‐CoV‐2 infection: ↑Firmicutes/Bacteroidetes ratio Bacteroidetes ↓ (during recovery Bacteroidetes↓)
28	^62^	USA	2021	Cross‐Sectional	*N* = 84 (48−70 years old)	Nasopharyngeal	16 S rRNA Amplicon Sequencing		↑Cyanobacterial ↑Cutibacterium ↑Lentimonas ↓Prevotellaceae ↓Luminiphilus ↓Flectobacillus ↓Comamonas ↓Jannaschia	nasopharyngeal: ↑Cyanobacterial in COVID + patients. Symptomatic COVID patients had ↑Cutibacterium ↑Lentimonas than asymptomatic patients. Dysbiosis + (May have a relation to COVID severity). Changes in microbiota may have immunogenic effects.
29	^63^	China	2021	Cohort	*N* = 66	Gut	Shotgun Metagenomic Sequencing	Associations: ALT, RBC, hemoglobin level ~Coprococcuscatus. AST~Streptococcus salivarius. RBC level~ Eubacterium hallii. Neutrophil ~Clostridium nexile,	↑Bacteroides stercoris, Bifidobacterium longum, Streptococcus thermophilus, Lachnospiraceae bacterium 5163FAA, ↓Clostridium nexile, Streptococcus salivarius, *Enterobacter aerogenes*, ↓Candidatussaccharibacteria	Changes in gut microbiota can change the course and severity of COVID‐19 disease ↓Microbiota variation ↑Bacteroidetes/Firmicutes ratio
30	^64^	China	2021	Cross‐sectional	*N* = 39	Sputum	Oxford Nanopore Technology sequencing platform		Severe COVID: ↓Neisseria, Rothia, Prevotella	Characteristics of sputum microbiota are variable in different COVID‐19 severity stages. After recovery, their microbiota becomes near similar to that of healthy individuals
31	^33^	China	2021	Interventional	*N* = 11 median age: 49	‐	Fecal microbiota transplantation (FMT); 10 capsules each day for 4 consecutive days.	After using FMT: microbial richness↑ alpha diversity ↔	‐	Using FMT consequences: ↓naive B cell ↑memory B cells ↑non‐switched B cells Restore the gut microbiota as: ↑Actinobacteria (15.0%) ↓Proteobacteria (2.8%) ↑Bifidobacterium ↑Faecalibacterium Palliate GI symptoms
32	^65^	China	2021	Cohort	*N* = 15 27−76	Nasopharynx Urine Serum	Leptotrichiahofstadii Gemellamorbillorum Gemellahaemolysans Streptococcus sanguinis Veillonelladispar Prevotellahisticola	Increased Leptotrichiahofstadii and Gemellahaemolysans in nasopharyngeal microbiome Is linked to CME levels in serum. CME seems to be helpful to treat COVID‐19.	The nasopharyngeal microbiome of COVID‐19 patients: Leptotrichiahofstadii↓ Gemellamorbillorum↓ Gemellahaemolysans↓ Streptococcus sanguinis↑ Veillonelladispar↑ Prevotellahisticola↑	Serum of COVID‐19 patients: Chlorogenic acid methyl ester (CME) ↓ Lactic acid↓ l‐Proline↓
33	^32^	Belgium	2021	Cohort	*N* = 93 Upper respiratory = 61 (37–83) Lower Respiratory = 64 (45–85)	Respiratory tract		Some bacteria in the respiratory tract can lead to immune reactions.		Duration of hospitalization in ICU and type of oxygen therapy have higher impacts on microbiota composition than the viral load of COVID‐19.
34	^49^	China	2021	Cohort	*N* = 88 Median age: 50	Oropharynx	Rothia Pseudopropionibacterium Streptococus Veillonella Megasphaera veilonella	Changes in microbiota can be linked to immune responses and the severity of the disease. Some pathogens(Klebsiella and Serratia) were linked to more severe diseases.	Microbiota of COVID‐19 patients was changed notably. (Diversity↓ beneficial bacteria↓ Opportunistic pathogens ↑ )	In COVID‐19 patients: Rothia↓ Pseudopropionibacterium↓ Streptococcus↓ Veillonella ↑ (most specific for COVID‐19) Megasphaera↑
35	^54^	Pennsylvania (USA)	2021	Cross‐sectional	*N* = 96 Median Age (COVID‐19 group):36−91 Non‐COVID = 60 (39–94)	Nasopharynx Oropharynx Endotracheal aspirate	Staphylococcus Redondoviridae Anellovirdae	The composition of the microbiota is linked to Lymphocyte/neutrophil (ratio) and consequently, it is linked to the severity of the disease.	The microbiota of the Respiratory tract in COVID‐19 patients had notable differences in comparison with patients who had other severe diseases.	In intubated COVID‐19 patients: Staphylococcus↑ Redondoviridae↑ Anellovirdae↑
36	^34^	Russia	2021	Prospective Cohort	*N* = 100 Age:18−60		Lactobacillus plantarum Bifidobacterium bifidum	In this study administration of a probiotic formula in COVID‐19 patients improved the weakness and shortened the diarrhea duration.		
37	^68^	China	2021	Cohort	*N* = 323 Median age = 70.5 (25−88)		Acinetobacter klebsiella			The study reported that changes in airway microbiota in severe COVID‐19 patients may be due to intubation.
38	^69^	USA	2021	Cohort	*N* = 112 Mean age = 56	Saliva	16 S rRNA sequencing Streptococcus, Prevotella	‐	Alpha and Beta diversity:no significant change In COVID‐19 patients: ↑Prevotellapallens ↓Rothiamucilaginosa ↓Streptococcus spp	Only a mild difference between the saliva microbiome of the COVID‐19 and healthy individuals was seen.
39	^56^	Portugal	2021	Cross‐sectional	*N* = 115, Median age: 68.0 (52.0–76.0)	Gut	Proteobacteria Roseburia Lachnospira	It seems that Gut microbiota composition can be a predictive factor for the severity of COVID‐19 disease.	Severe and moderate COVID‐19 patients had a remarkable change in Gut microbiome composition.	Gut microbiota in moderate and severe COVID‐19 patients: Roseburia (butyrate‐producing) ↓ Lachnospira (butyrate‐producing) ↓ Proteobacteria ↑
40	^71^	Italy	2021	Cross‐sectional	*N* = 38, Age (COVID‐19 group): 35−84	Nasopharynx	Fusobacterium Periodonticum		The nasopharyngeal microbiome of COVID‐19 patients was notably changed compared to Healthy persons.	The study suggests that the remarkable depletion of Fusobacterium Periodonticum may be due to its surface sialylation ability.
41	^72^	Mississippi (USA)	2021	Cohort	*N* = 93 Mean age COVID‐19 patients:62.3 ± 13.4 Recovered patients:46.7 ± 16.1	Gut	Campylobacter Corynebacterium Klebsiella	Due to this study the composition of the gut microbiome is not related to the severity of the disease.	the gut microbial composition in COVID‐19 patients is notably changed in comparison with healthy individuals. The recovered patients’ gut microbial composition is similar to the control group.	Gut microbiome of COVID‐19 patients: campylobacter↑ corynebacterium↑
42	^73^	Portugal	2021	Observational					social distancing during lockdown: ↓bacterial transmission between people, leading to ↓antibiotic consumption. antibiotic resistance genes in the microbiome ↓	
43	^74^	Germany	2021	Cohort	*N* = 212, Mean age in COVID‐19 group = 56 ± 19	Gut	Streptococcus Bifidobacterium Collinsella Roesburia (butyrate‐producing) Faecalibcterium (butyrate‐producing)	Reduced butyrate‐producing bacteria in the gut microbiome are linked to severe disease.	The gut microbiome of COVID‐19 patients had a much more depleted bacterial richness.	Gut microbiome of COVID‐19 patients: Streptococcus↓ Bifidobacterium↓ Collinsella↓
44	^16^	China	2021	Cross‐Sectional	*N* = 192 Age: 49−68	Oropharynx	Streptococcus Serratia Candida Enterococcus	there is a notable link between URT microbiota and inflammatory Cytokine levels and therefore disease severity/mortality.	Microbiota of the upper respiratory tract in COVID‐19 patients was different in comparison with healthy individuals.	Streptococcus was found in abundance in the URT microbiota of recovered patients. Candida and Enterococcus were detected in abundance in the URT microbiota of deceased COVID‐19 patients.
45	^75^	USA	2021	Cross‐ sectional	‐	‐	‐	Gut microorganisms’ impact on ACE2 and TMPRSS2 may influence the risk of SARS‐CoV‐2 infection. The gut microbiota activating MAIT cells, influence COVID‐19 severity by affecting T and B cell function. Inflammation in autoimmune disorders and COVID‐19 may be exacerbated by gut barrier impairment.	The SARS‐CoV‐2 spike protein binds directly to LPS, altering its function and aggregation state, hence increasing pro‐inflammatory activity.	The gut microbiome is vital in controlling and training the host's immune system.
46	^78^	Italy	2021	Cross‐sectional observational Study	39 COVID‐19 patients Mean age = 71.1 ± 18.4 years	Oral	Streptococcus, Veillonella, Prevotella, Lactobacillus, Capnocytophaga, Abiotrophia, Aggregatibacter, Atopobium,	Streptococcus↑, Veillonella, Prevotella↑, Lactobacillus↑, Capnocytophaga↑, Abiotrophia↑, Aggregatibacter↑, Atopobium↑, Haemophilus↓, Parvimonas↓,	With COVID‐19, significant drop in alpha‐diversity and bacteria species richness, with a strong link between these decreases and symptom intensity with an increase of pro‐inflammatory cytokines like IL‐6, TNFa, and IL‐1b.	The oral microbiome's fungal component showed significant variances. COVID‐19 patients had a higher oral virome than controls. TNFa and GM‐CSF concentrations were higher in COVID‐19 patients, but not statistically significant.
47	^35^	Russia	2021	Cross‐sectional	‐	‐	Probiotic bacteria, Lactobacillus plantarum, Bifidobacterium bifidum	Probiotic Lactobacillus strains produce organic acids, ethanol, and exopolysaccharides, all of which have antiviral effects. The Bifidobacterium genus produces organic acids, ethanol, exopolysaccharides, and cell wall‐released lipoproteins, which can block viral particle interactions with human mucous membrane receptors, halting infection progression.	‐	Bacterial probiotics prevent respiratory virus proliferation in cell culture.
48	^36^	USA	2021	Clinical trial protocol	*N* = 1132 Age ≥ 1 year Children	Nasal swabs, stool samples	Lactobacillus rhamnosus GG	Taking LGG as a probiotic will protect against SARS‐CoV‐2 infection and reduce the severity of disease, and will be associated with beneficial changes in the composition of the gut microbiome.	‐	Impact of LGG on the microbiome in SARS‐CoV‐2 infection, symptomatology, and clinical complications; differences in baseline microbiome predicting COVID‐19 infection (ie, protective microbiome signature); effect of SARS‐CoV‐2 infection on changes in microbiome; the impact of LGG on the microbiome in EHC at high risk of COVID‐19 disease.
49	^79^	China	2021	Cross‐sectional	7 recovered COVID‐19 male patients, 3‐months after discharge.	Fecal	‐	Rothia↑ Erysipelatoclostridium↑ Streptococcus, Actinomyces, and Veillonella increases were noted but not statistically significant. anti‐inflammatory bacteria↓	‐	The gut microbiota of recovered patients varied from healthy controls in terms of Chao index, Simpson index, and b‐diversity. The unbalanced gut flora may not be totally repaired in recovered COVID‐19 patients.
50	^81^	Spain	2020	Retrospective cohort	*N* = 177 median age of 68.0 years	Nasopharyngeal	Actinobacillus spp., Citrobacter spp., Craurococcus spp., or Moheibacter spp.	‐	Reduce the risk of IMV and reduce the risk of death	The microbial αdiversity indexes were lower in patients who died, and the βdiversity analysis revealed considerable clustering. A more diverse nasopharyngeal microbiota with certain species seems to be an early biomarker of clinical improvement in hospitalized COVID‐19 patients.
51	^37^	China	2021	Randomized controlled trial	Patients with mild‐to‐severe COVID‐19 and suspected GMD.	Nasopharyngeal swab, feces	‐	‐	‐	The impact of WMT on organ function, homeostasis, inflammatory response, intestinal mucosal barrier function, and immunity in COVD‐19 patients suspected of having GMD. WMT is effective and safe for COVID‐19 patients.
52	^15^	China	2021	Cross‐Sectional	53 COVID‐19 patients	Throat swabs, fecal	‐	Blautia↓, Coprococcus↓, Collinsella↓, B. caccae↓, B. coprophilus↓C. colinum species↓; Streptococcus↑, Enterococcus↑, Lactobacillus↑, Actinomyces↑, Granulicatella ↑at the genus level, C. citroniae↑, B. longum, R. mucilaginosa↑	Neisseria↓ Corynebacterium↓, Actinobacillus↓, Moryella↓, Aggregatibacter↓, Treponema↓, and Pseudomonas↓ at the genus level, *P. intermedia*↓ Veillonella↑, Campylobacter↑, Kingella↑, H. parainfluenzae↑, R. mucilaginosa↑, N. subflava↑	The alpha and beta diversity indexes showed that SARS‐CoV‐2 infection altered the microbiome community in patients.
53	^82^	China	2021	Cross‐ sectional	11 COVID‐19	Pharyngeal swabs	‐	Streptococcus suis and *S. agalactiae* might induce ACE2 expression in Vero cells, promoting SARS‐CoV‐2 infection. These enhanced pathogens in pharynxes may produce secondary bacterial infections by altering the expression of the viral receptor ACE2 or modulating the host's immune system.	‐	COVID‐19 enhanced pathogens may play a role in SARS‐CoV‐2 infections. The alpha diversity of the two patient samples (COVID‐19 and non‐COVID‐19) differed significantly from the healthy individual group. Observed species and Shannon index showed no significant difference.
54	^83^	China	2021	Cross‐ sectional	9 COVID‐19 children, (7−139 months)	Throat swabs, nasal swabs, or feces	‐	Bacteroidetes↑, Firmicutes↑ Proteobacteria↑ in the respiratory tract Bacteroidetes↑, Firmicutes ↑ in the gut. Pseudomonas↑, in both the upper respiratory tract and the gut Comamonadaceae_U↑ in the upper respiratory tract	The microbiomes in COVID‐19 children's throat and nasal swabs were considerably less rich And the gut microbiota was found to be more even than that of healthy controls.	SARS‐CoV‐2 infection changes upper respiratory tract and gut microbiomes in nine children.
55	^84^	China	2021	Cohort	*N* = 100, 36.4 ± 18.7	Gut	Eubacterium rectale Bifidobacteria Faecalibacterium prausnitzii Bacteroides dorei	The composition of gut microbiota in COVID‐19 patients is notably linked to the level of inflammatory cytokines and severity of the disease. Lasting gut microbiota changes in COVID‐19 patients after recovery leads to persistent symptoms.	Gut microbiota is meaningfully changed in COVID‐19 patients.	Gut microbiota in COVID‐19 patients: Eubacterium rectale↓ Bifidobacteria↓ Faecalibacterium prausnitzii↓ Bacteroides dorei↑
56	^85^	China	2021	Cross‐sectional	*N* = 66, Mean = 42.6 ± 19	Gut	Bifidobacterium adolescentis F prausnitzii Ruminococcus bromii Bacteroides dorei Bacteroides ovatus Bacteroides thetaiotaomicron	The microbiota changes in COVID‐19 patients lead to increased symptoms and more severe disease.	The gut microbiota of COVID‐19 patients, (especially in severe disease) changed meaningfully compared to healthy individuals. Bifidobacterium↓ F prausinitzii↓	The changes in the microbiota in COVID‐19 patients lead to Lower levels of l‐Isoleucine and SCFA (Short‐Chain Fatty Acid) and l‐Isoleucine even one month after recovery and this causes more severe disease.
57	^38^	China	2021	Cohort	*N* = 375 Median age = 50 (Nonprobiotic) 48 (Probiotic)	Gut	Lactobacillus, Bifidobacterium Enterococcus	Probiotics reduced the length of COVID‐19 illness and hospitalization.		Administration of probiotics enhanced the condition of COVID‐19 patients.
58	^39^	China	2022	Clinical Trial	*N* = 55	Gut	Bifidobacteria	Administration of SIM01 (a microbiome compound) in COVID‐19 patients led to increased antibodies and lower levels of inflammatory markers.		
59	^86^	China	2021	Cross‐sectional	*N* = 187 Mean age: 39 (32–57)	Gut	*Saccharomyces cerevisiae* Enterococcus faecalis *Bacteroides fragilis*	The gut microbiota in COVID‐19 patients with fever was different from those without fever. it seems that the gut microbiota changes can play a part in causing fever through inflammatory reactions.		In COVID‐19 patients with fever: *Saccharomyces cerevisiae*↑ Enterococcus faecalis↑ COVID‐19 patients without fever: *Bacteroides fragilis*↑
60	^87^	China	2021	Cohort	*N* = 29 Age: 28−41 Median: 29	Gut	F prausnitzii Escherichia unclassifies	The lasting gut microbiota dysbiosis of healthcare workers 3 months after recovery leads to persistent symptoms.	The Gut microbiota of Healthcare workers with previous SARS‐CoV‐2 infection was different in comparison to non‐COVID group even 3 months after recovery. (beneficial bacteria↓ Opportunistic pathogens ↑)	
61	^67^	China	2021	Pilot observational study	*N* = 15, Mean= 53.8	Gut	Morganellamorgani Collinsella aerofaciens Streptococcus infantis		In COVID‐19 patients, the gut microbiota was changed and opportunistic pathogens were increased.	Gut microbiota in COVID‐19 patients: Morganellamorgani↑ Collinsella aerofaciens↑ Streptococcus infantis↑
62	^88^	China	2020	Cross‐scectional	*N* = 69, Median Age: 46 (COVID‐19) 63 (Pneumonia) 34 (Healthy)	Gut	Aspergillus flavus *Candida albicans* Candida auris		In COVID‐19 patients, the gut microbiome was different in comparison with the non‐COVID group. Candida species↑	In COVID‐19 patients Aspergillus flavus, *Candida albicans*, and candida Auris were increased in the gut microbiome and they were not found in healthy individuals
63	^80^	China	2020	Cross‐sectional	*N* = 36, Median Age: 55 (COVID +) 50 (Pneumonia +) 48 (Healthy)	Gut	Coprobacilum Clostridium ramosum Clostridium hathewayi F prausnitzii	The changes in the gut microbiome of COVID‐19 patients can cause more severe disease.	The gut microbiome was different in COVID‐19 patients compared to non‐COVID group. (beneficial bacteria↓ Opportunistic pathogens↑)	Coprobacilum, ramosum Clostridium, ramosum and Clostridium hathewayi were linked to more severe disease, while F prausnitzii has a negative correlation to the severity of the disease.

**Table 2:** Newcastle−Ottawa Scale (NOS) bias risk assessment of the study.

Reference	Selection (out of 4)	Comparability (out of 2)	Exposure/outcome (out of 3)	Total (out of 9)
^29^	3	1	2	6
^23^	3	2	2	7
^30^	3	2	2	7
^31^	2	2	3	7
^32^	3	2	3	8
^33^	3	1	2	6
^28^	4	2	3	9
^34^	3	1	3	7
^35^	3	1	3	7
^36^	3	1	3	7
^24^	2	2	1	5
^37^	2	1	2	5
^38^	3	2	2	7
^39^	3	2	3	8
^40^	3	1	2	6
^41^	2	2	3	7
^42^	2	1	2	5
^43^	4	1	2	7
^44^	4	1	2	7
^45^	3	2	2	7
^21^	3	2	2	7
^20^	3	1	2	6
^46^	3	1	2	6
^47^	3	1	2	6
^48^	3	2	2	7
^49^	3	1	1	5
^50^	4	1	3	8
^51^	3	2	3	8
^52^	3	2	2	7
^53^	2	2	2	6
^54^	2	2	2	6
^55^	3	2	2	7
^22^	3	2	2	7
^25^	2	2	2	6
^26^	4	1	2	7
^56^	3	1	3	7
^57^	3	1	2	6
^58^	3	1	3	7
^27^	3	2	3	8
^59^	4	1	2	7
^60^	3	2	3	8
^61^	4	2	2	8
^62^	4	2	2	8
^63^	3	2	2	7
^64^	3	2	2	7
^65^	3	2	2	7
^66^	4	2	2	8
^67^	3	2	2	7
^68^	3	1	2	6
^69^	3	2	2	7
^70^	3	1	3	7
^71^	3	1	3	7
^72^	3	2	3	8
^73^	4	2	2	8
^74^	4	2	3	9
^75^	4	2	2	8
^76^	3	2	2	7
^77^	3	1	3	7
^78^	3	1	2	6
^79^	3	2	3	8
^80^	4	2	2	8
^81^	3	1	2	6
^20^	3	1	2	6

## 3 RESULTS

A total of 829 articles were collected in this systematic review. After the duplicate removal, 508 publications were selected based on the relevancy of the title and abstract, and 293 articles were excluded in this step. An additional 152 articles were excluded in the full‐text screening, and 63 articles were included in the final qualitative synthesis (Figure 1).

**Figure 1:** PRISMA flow diagram of the study selection process. PRISMA, Preferred Reporting Items for Systematic Reviews and Meta‐Analyses.

Most of the studies were conducted in 2020 (9.52%) and 2021 (88.8%). One study was carried out in 2022. China (25 articles) and the United States (11 articles) accounted for the source of the majority of included studies. Six articles were from Italy, three studies were from Russia, and the remaining was from other countries. In most of the articles, samples were collected from the gut and the other studies examined the microbiota of the oropharynx, nasopharynx, respiratory tract, sputum, saliva, and blood. One study evaluated the microbiome in the waste water.

Most articles claimed that SARS‐CoV‐2 infection causes microbiome disbyosis in the patients. Zuo et al., reported that the Gut microbiome in COVID‐19 patients was meaningfully different compared to non‐COVID group with an increase in opportunistic pathogens and a decrease in beneficial bacteria.^80^ According to Hernández‐Terán et al. the respiratory microbiome of COVID patients has a high level of dysbiosis, while Miller et al claimed that there was no notable difference in saliva microbiota of COVID‐19 patients in comparison with healthy individuals.^31^ Lloréns‐Rico et al. suggested that duration of hospitalization in ICU and type of oxygen therapy have higher impacts on the composition of respiratory tract microbiota than the viral load of COVID‐19.^32^

The composition of microbiota may also be linked to the severity of COVID‐19 disease according to the majority of the articles.^45^, ^48^, ^49^, ^54^, ^56^ It appeared that COVID‐19 patients with severe disease had more dysbiotic microbiota. An increase in Firmicutes/Bacteroidetes ratio was also observed in some studies. Several studies reported that the changes in the microbiota of COVID‐19 patients can last even for a period after recovery.^66^, ^67^

Some articles also evaluated the effect of probiotics on SARS‐CoV‐2 infection. The majority of the studies found the probiotics beneficial for COVID‐19 patients’ recovery.^29^, ^30^, ^33^, ^34^, ^35^, ^36^, ^37^, ^38^, ^39^, ^45^, ^70^, ^76^, ^77^ One study evaluated the positive efficacy of FMT (Fecal microbial transplantation) for COVID‐induced GI upset.^33^ Zhang et al. reported that probiotics reduced the length of COVID‐19 illness and hospitalization.^38^ In contrast, Ivashkin et al. evaluated a probiotic formula and suggests that the tried probiotic had no noteworthy impact on the severity of the disease or mortality in COVID‐19 patients.^29^ Hegazy et al. reported that intake of probiotic yogurt is linked to a notable higher risk of severe SARS‐CoV‐2 infection.^77^

43 publications out of the 63 total articles considered in this systematic review, studied the impact of SARS‐CoV‐2 infection on the microbiota. The effect of SARS‐CoV‐2 infection on microbiota and vice versa was studied in 21 articles, and 20 publications investigated the effect of either microbiota profile or various probiotics on the course of COVID‐19 disease.

## 4 DISCUSSION

### 4.1 Gut microbiome dysbiosis of COVID‐19 patients

Dysbiosis in the gut‐lung axis can cause a proinflammatory reaction.^89^, ^90^ Additionally, it is shown that gut dysbiosis has a role in the pathogenesis of several diseases including; IBD, Parkinson's disease, celiac disease, diabetes, colorectal cancer, and chronic respiratory diseases like COPD, and Asthma.^91^, ^92^, ^93^, ^94^, ^95^, ^96^ Many studies have reported gut dysbiosis among COVID‐19 patients and noted that it would be a major contributor to poor outcomes.^97^

The majority of human gut bacteria comprise the following microbial phyla; *Firmicutes, Bacteroidetes, Actinobacteria, Proteobacteria, Fusobacteria*, and *Verrucomicrobiac* with *Firmicutes* and *Bacteroidetes* making up over 90% of the total gut microbiota.^98^, ^99^, ^100^ These bacteria can regulate and control the immune response and defense system via a variety of mechanisms, and any imbalance in their composition can lead to immune dysfunction and pathogenesis.^101^, ^102^

Gut dysbiosis has been reported in almost all included studies in our systematic review, and in total 25 studies, investigated the two‐way dynamics between COVID‐19 and gut microbiota mostly via fecal/colon sampling.

In general, the main alternations in the gut microbiome of COVID‐19 cases compared to normal conditions were the higher abundance of *Bacteroides, Streptococcus, Fusobacterium, Campylobacter, Lactobacillus, Proteobacteria, Enterococcaceae, Enterococcus, Rothia, Pseudomonas, Veillonella, Clostridium*, and *Staphylococcaceae*, and lower presence of *Coprococcus, Faecalibacterium, Eubacterium, Roseburia, Bifidobacterium*, and *Blautia*.

### 4.2 Specific differences in gut microbiome of COVID‐19 patients compared to the general healthy population

Five included studies reported an increase in *Bacteroides* in COVID‐19 patients^51^, ^63^, ^84^, ^85^, ^86^ while only one reported a decrease.^40^ These studies observed a rise in *Bacteroides stercoris, Bacteroides dorei, Bacteroides vulgatus, Bacteroides massiliensis, Bacteroides oleiciplenus*, and *Bacteroides ovatus* as main species in fecal samples of COVID‐19 patients. Additionally, one study reported an increase in *Bacteroides fragilis* in afebrile COVID‐19 patients. *Bacteroides* have a crucial role in the gut microbiome and their alterations have been linked to several diseases.^103^, ^104^, ^105^ Additionally, it is shown that*Bacteroides* could downregulate ACE‐2 receptor expression^106^; thus, they probably can limit SARS‐CoV‐2 replication in the gut. *Bacteroides dorei* is a controversial bacterium because of the fact that they also can downregulate the ACE‐2 receptor but they are also linked to some proinflammatory cytokines.^107^

One study reported a decrease in the levels of *Blautia spp*.,^15^ while another study reported increasing patterns.^40^ Also,*Blautia spp*. in the gut microbiome of CRC patients has been linked to more severe disease^42^ and its increased levels have been reported after COVID‐19 recovery.^44^ A similar study has reported increasing levels of opportunistic pathogens such as*Blautia spp*., and linked this species with a more severe illness.^108^

One study reported decreasing levels of *Clostridium nexile*,^63^ and another article reported possible associations between*Clostridium ramosum and Clostridium hatheway* with severe forms of COVID‐19 disease and portal vein thrombosis.^80^ Also,*Clostridium leptum* has been positively correlated to neutrophil counts in COVID‐19 patients; while *Clostridium butyricum* is negatively correlated.^36^ Some studies have also reported that increasing levels of *Clostridium difficile* can worsen COVID‐19 patients' condition.^109^, ^110^

Four studies reported increasing levels of *Streptococcus spp*.^40^, ^63^, ^67^, ^79^ and two articles specified *Streptococcus thermophilus*,^63^ and *Streptococcus infantis* ^67^ as the main increasing bacteria, while two studies reported its decreased levels.^63^, ^74^ Some studies have noted the increase in*Streptococcus spp*. would be an indicator of opportunistic pathogens abundance.^111^, ^112^ *Streptococcus* increase has been linked to the excessive expressions of proinflammatory cytokines.^112^, ^113^ *Streptococcus thermophilusis* was also positively correlated with the severity of COVID‐19.^63^ It is also shown that*Streptococcus spp*. can impact the lung microbiome and cause inflammatory conditions.^114^

One study reported an increase in *Lachnospira* levels^63^ while the other study reported a decline in its levels.^56^ Several studies have reported that*Lachnospira* assists with gut homeostasis among COVID‐19 patients.^105^, ^115^, ^116^, ^117^

Two articles reported a declining pattern of *Coprococcus genus* in the gut microflora of COVID‐19 patients.^15^, ^63^ Cao et al. showed that*Coprococcus catus* could decrease among antibiotic‐receiving COVID‐19 patients.^115^ In addition, one study found relatively lower levels of *Coprococcus*, in COVID‐19 patients compared to both flu patients and healthy cases.^112^ *Coprococcus* was also reported to be positively correlated with lymphocyte counts.^118^

Regarding *Eubacterium, Eubacterium hallii* and *Eubacterium rectale* were the main species that declined.^63^, ^84^ Many other studies have reported its decreasing levels can be linked to antibiotic overuse among COVID‐19 patients.^106^, ^119^ While, *Eubacterium ventriosum* have been shown to have anti‐inflammatory effects.^115^

*Fusobacterium ulcerans* was unique bacteria found in COVID‐19 patients' microflora.^63^ It has been found that the abundance of *Fusobacterium* would increase proinflammatory factors.^120^

Two studies reported increasing levels of *Campylobacter*,^15^, ^72^ and one study found possible associations between this genus with a more severe disease.^48^ One similar study has reported the abundance of *Campylobacter gracilis* among severe cases of COVID‐19.^115^ Also, one study has mentioned*Campylobacter* among the top three abundant opportunistic pathogens.^82^

One study reported an increase in *Corynebacterium* levels,^72^ while one other study reported a decrease.^15^ In a similar study, *Corynebacterium durum* was reported to be increased among severe COVID‐19 cases.^115^

Four studies stated a decrease in *Bifidobacterium* in COVID‐19 patients' gut microbiome^40^, ^74^, ^84^, ^85^ while only one study reported an increase in its levels.^63^ Many species of these genera including; *Bifidobacterium animalis, B. longum* and *B. bifidum* have been shown to reduce the levels of inflammatory cytokines, and enhance anti‐inflammatory cytokines.^121^ In addition, the scientific society has a particular interest in this bacterium as a probiotic with anti‐inflammatory properties for the treatment of many conditions ranging from IBD to *Clostridioides difficile* infection.^122^, ^123^ Similar studies also reported a decline in *Bifidobacterium* of COVID‐19 patients' gut microbiome.^124^ This shows the possible vital effects of this genus in regulating the immune system and outlines that its decline among COVID‐19 patients would have detrimental impacts on the prognosis and severity of the disease.

Two studies reported *Lactobacillus* increase.^50^, ^85^ While one study reported a decline in*Lactobacillus spp*. in the samples of COVID‐19 patients.^125^ One similar study conducted in China reported decreased levels of *Lactobacillus*.^126^ It has been shown that gut commensals including*lactobacillus* regulate the immune system, and *Lactobacillus casei* would enhance the phagocytic activity of macrophages and has protective effects against flu virus infections. These studies signify the possible anti‐inflammatory effects of *Lactobacillus*.^127^

*Roseburia* decrease was reported and linked to severe COVID‐19 infection.^56^ Similar studies showed*Roseburia* decrease among COVID‐19 and influenza cases.^80^, ^89^, ^115^, ^128^ *Roseburia* is anti‐inflammatory, maintains mucosal integrity, limits the opportunistic pathogens’ overgrowth, and improve antiviral immunity.^129^, ^130^ Thus, its possible decrease in COVID‐19 patients would probably predispose them to a more severe disease course.

One study has reported a decline in *Faecalibacterium prausnitzii*,^84^ while another study reported an increase in this genus.^40^ Similarly, a significantly lower abundance of *Faecalibacterium* among COVID‐19 patients was reported by Hazan et al., who also reported that the increase of *Faecalibacterium prausnitzii* was inversely associated with SARS‐CoV‐2 positivity and COVID‐19 severity.^124^ In addition, many studies have linked*Faecalibacterium* decrease to COVID‐19 severity.^36^, ^114^

One study reported that *Firmicutes* was observed more among negative or recovered COVID‐19 patients^44^ and two studies reported declining patterns of this bacteria^50^, ^57^ while, two other studies reported its increasing levels.^61^, ^83^ In addition, one study has shown that the*Firmicutes* to *Bacteroidetes* had increased among acute COVID‐19 patients.^61^ Conversely, another study reported the opposite and stated that this ratio had declined among them.^63^ Khan et al. also reported significant decrease in *Firmicutes* among COVID‐19 patients, and also indicated a gradual decline in *Firmicutes* to *Bacteroidetes* ratio from mild to severe COVID‐19 infected groups,^116^ similarly this decline has been reported in systemic inflammation, cognitive disorders, Crohn's disease, depression, and diabetes mellitus type 2.^131^, ^132^ All these studies show the possible effects of *Firmicutes* and *Firmicutes* to *Bacteroidetes* ratio, on inflammatory and autoimmune reactions in a variety of diseases such as COVID‐19.

Three studies demonstrated *Enterococcaceae* and *Enterococcus* abundance in COVID‐19 patients' gut samples.^15^, ^50^, ^86^ Zou et al. specified*Enterococcus faecalis* as the main increasing species patients with fever.^86^ Tang et al. also stated that*Enterococcus* to *Enterobacteriaceae* ratio could change in severe/critical COVID‐19 cases, and it significantly rose in deceased patients compared to survivors, thus this index can have a predictive value for ill COVID‐19 patients.^133^ *Enterococcus* abundance may play an important role in the severity and poor outcomes of COVID‐19 patients.

*Rothia spp*. increase was reported by two studies.^15^, ^79^ Similarly, other studies have reported increasing levels of opportunistic bacteria including*Rothia spp*. among COVID‐19 patients.^79^, ^89^ Some studies have previously reported possible associations of this bacterium with lung injuries.^17^, ^106^ One study reported that*Rothia* was higher even among recovered patients compared to the control group, which would be indicative of COVID‐19 long‐term effects on gut microbiota.

One study reported a decrease in *Pseudomonas* levels^15^; while another study reported the opposite.^83^ Prasad et al. also reported an abundance of *Pseudomonas spp*. in blood samples of COVID‐19 patients.^125^ Pseudomonas was among the most predominant genera in the lung microbiome of COVID‐19 patients.^134^, ^135^

*Collinsella aerofaciens* was reported by one study to increase in gut microbiota,^67^ while other studies stated that it had decreasing patterns.^15^, ^74^ *Collinsella*, is reported by some studies in the gut microbiome of severe cases of COVID‐19 patients. One study reported that this bacteria has the following effects: limiting SARS‐CoV‐2 attachment to ACE‐2, suppressing inflammatory cytokines, and has antiapoptotic and antioxidant features, the same study concluded that lower presence of *Collinsella* was associated with high COVID‐19 mortality while its normal presence was significantly correlated to lower mortality rates among COVID‐19 patients.^136^

In regard to *Ruminococcus* genus, one study reported increasing levels of this bacteria in the gut flora of CRC patients that would predispose them to more severe COVID‐19 disease,^42^ and another study found a negative association between this bacteria and COVID‐19 viral load.^15^ Similar studies have reported a high abundance of *Ruminococcus gnavus*, and *Ruminococcus torques* species among COVID‐19 patients.^84^ Some studies have reported decreasing levels of *Ruminococcus bromii*, and *Ruminococcus obeum* in the gut flora of COVID‐19 patients.^80^, ^137^

One study had reported increasing levels of fungal microorganisms including; *Aspergillus flavus, Aspergillus niger*, and *Candida Albicans* in the gut microbiome of COVID‐19 patients.^88^ On the other hand, the study by Lv et al. reported a decrease in *Aspergillus rugulosus, Aspergillus tritici, and Aspergillus penicillioidein* COVID‐19 patients' gut microbiome.^137^

*Veillonella* genus increase among COVID‐19 patients was reported by three articles.^15^, ^50^, ^79^ Similar studies have reported the abundance of this bacterium in the gut microbiome composition of COVID‐19 patients, and one specified *Veillonella parvula* as the main increasing species.^89^, ^115^, ^138^ One study also indicated that *Veillonella* may be associated with the severity of COVID‐19.^138^

One study linked *Staphylococcus epidermis* with a more severe course of diseases,^48^ and another study reported its increasing levels in gut microbiota.^50^ Similarly, one study reported the abundance of *Staphylococcaceae spp*. in serums samples of COVID‐19 patients.^125^

### 4.3 URT microbiome dysbiosis of COVID‐19 patients

The relation between the microbiota of the URT, including nasopharyngeal, oropharyngeal, and respiratory tract, and COVID‐19 as a viral respiratory disease is an intricate, two‐sided, and dynamic association. In the current review, 24 studies discussed the possible role of URT microbiota alterations in the pathogenesis, and prognosis of COVID‐19 infection. The impact of URT microbiota on the preservation of the lung immune system is one of the important aspects as it correlates with respiratory infections.^43^, ^81^, ^139^ Unusual changes in URT microbiota in COVID‐19 patients, especially moderate and severe patients, were reported in comparison to healthy individuals.^31^, ^43^ The richness of microbiota was higher in COVID‐19 patients^59^, ^78^ and most of them were opportunistic bacteria.^58^ COVID‐19 infection would possibly induce URT microbiota to multiply the inflammatory bacteria like *Haemophilus influenzeae* and *parainfluenzae* which are associated with acute respiratory diseases like pneumonia.^43^ Also, it may increase *Neisseria subflava*; which its decrease in COVID‐19 patients was significantly related to a high rate of mortality.^31^, ^43^ The high level of *Klebsiella* and *Serratia* were also associated with more severe diseases.^140^

We found that the duration of hospitalization in ICU and the type of oxygen therapy have a higher impact on the composition of microbiota compared to SARS‐CoV‐2 viral load.^32^, ^55^ Certainly, microbiome dysbiosis (Bacteria, viruses, and archaea) can cause an abnormal inflammatory response that could lead to poorer COVID‐19 outcomes.^58^ A notable association between URT and inflammatory cytokines levels (like IL‐6, TNF‐α, and IL‐1b) was observed and it can explain the significant link between URT microbiota and COVID‐19 severity and mortality rate.^16^, ^78^ These statements are consistent with the findings of some studies about the higher reduction of anti‐inflammatory metabolic factors in long COVID‐19 patients treated with antibiotics, invasive mechanical ventilation, and ICU admission compared to mild patients.^32^, ^43^, ^55^, ^141^ In addition, a quick return of dysbiosis level to normal values during recovery in mild COVID‐19 cases was reported.^20^, ^53^ Jing Liu et al. found that the microbiota level of COVID‐19 patients after recovery becomes near similar to that of healthy individuals.^141^

Some studies showed that the abundance and diversity of URT microbiota in severe and moderate COVID‐19 patients had no significant difference in comparison with mild COVID‐19 patients and healthy individuals.^20^ Also, the same diversity was reported in the analysis of specific kinds of microbiota; in microbial alpha‐diversity^46^, ^59^, ^69^, ^82^ and beta‐diversity.^69^, ^82^ In contrast, changes in microbial indices were reported by Ventero et al. as lower microbial alpha‐diversity and higher beta‐diversity among deceased COVID‐19 patients.^81^ Another study showed a significant reduction of taxonomic features richness in beta‐diversity in COVID‐19 patients.^46^ The findings of a study by the alpha‐diversity analysis for microbiome richness suggested that recovered patients had a higher diversity of microbiota than healthy individuals, and the healthy individuals had a higher diversity of microbiota compared with acute COVID‐19 patients.^58^ Accordingly, a more diverse URT microbiota seems to be an early biomarker of clinical improvement in COVID‐19 patients.^81^

### 4.4 Specific differences in URT microbiome of COVID‐19 patients compared to the general healthy population

Genus *Streptococcus* increases in COVID‐19 patients.^15^, ^16^, ^31^, ^46^, ^55^, ^65^, ^78^ The *Streptococcus* abundance is representative of opportunistic bacterial invasion extent.^112^ The abundance of *Streptococcus* is associated with higher expression of IFN‐ƴ, IL‐18, IL‐6, and TNF‐α and further inflammatory cytokines which worsens the clinical outcome of infection.^78^, ^112^, ^142^ The genus *Rothiais* widely found in the URT of patients with COVID‐19 infection.^15^, ^31^, ^46^, ^55^, ^62^ It seems that this genus is associated with lung injuries due to inflammatory activities.^55^, ^143^ The opportunistic pathogenic genus, *Corynebacterium*, is reported in COVID‐19 patients.^31^, ^59^ *Corynebacterium* is one of the microbiotas in URT whose alternation is associated with the severity of COVID‐19 and poor prognosis.^53^, ^59^ There is dominancy of genus *Prevotella* and *Veillonella* in COVID‐19 patients which could influence the progression of pneumonia.^31^, ^60^, ^65^, ^78^ These species could be associated with an increased risk of mortality in older and severe COVID‐19 patients due to pneumonia.^15^, ^55^, ^69^, ^140^

Other opportunistic pathogenesis of the URT like *Haemophilus, Stenotrophomonas, Acinetobacter, Moraxella, Corynebacterium, Gemella, Ralstonia, Pseudomonas*,^53^ *Granulicatella*,^52^ *Megasphaera* ^140^ were increased in COVID‐19 patients which are associated with serious clinical outcomes. Also, in severe COVID‐19 patients, an increase of *Megasphaera*, and infatal COVID‐19 patients increase *Rothiadentocariosa*, *Streptococcus infantis*, *Veillonelladispar* ^31^ were seen which may be associated with secondary pneumonia due to mechanical ventilation.

Finally, there is evidence that altered gut microbiota composition has a crucial role in the severity and virulence of many other bacterial and viral infections.^144^ Also, other studies have stated that the gut microbiota plays an important part in the pulmonary defense mechanisms against many respiratory infections including influenza A virus and respiratory syncytial virus infections.^145^ Thus the findings of this study, that the COVID‐19 is associated with gut‐lung microbiota differences compared to the general healthy population, are in line with other similar viral or bacterial infections (Table 3).

**Table 3:** A summary of associations between COVID‐19 and gut/upper respiratory tract microbiome.

Gut microbiota and COVID‐19 associations		
Family/genus/species	Number of studies that reported increasing patterns	Number of studies that reported decreasing patterns
Bacteroides	5	1
Blautia	1	1
Clostridium	‐	1
Streptococcus	5	2
Lachnospira	1	1
Coprococcus	‐	2
Eubacterium	‐	2
Fusobacterium	1	‐
Campylobacter	2	‐
Corynebacterium	1	1
Bifidobacterium	1	4
Lactobacillus	2	1
Faecalibacterium	1	1
Firmicutes	2	2
Enterococcaceae/Enterococcus	3	‐
Rothia	2	‐
Pseudomonas	‐	1
Collinsella	1	2
Ruminococcus	1	‐
Aspergillus/Candida	1	‐
Veillonella	3	‐
Staphylococcus	1	‐

Upper respiratory tract microbiota and COVID‐19 associations		
Family/Genus/Species	Number of studies that reported increasing patterns	Number of studies that reported decreasing patterns
Streptococcus	7	‐
Rothiais	5	‐
Corynebacterium	2	‐
Prevotella/Veillonella	4	‐
Haemophilus	1	‐
Stenotrophomonas	1	‐
Acinetobacter	1	‐
Moraxella	1	‐
Corynebacterium	1	‐
Gemella	1	‐
Ralstonia	1	‐
Pseudomonas	1	‐
Granulicatella	1	‐
Megasphaera	1	‐

## 5 ASSOCIATION BETWEEN COVID‐19 SEVERITY AND GUT MICROBIOME COMPOSITION

Five articles included in our study reported that gut microbiota composition can be a predictive factor in the severity of COVID‐19 disease.^48^, ^56^, ^63^, ^75^, ^84^ It has been shown that normal gut microbiota can decrease the severity of COVID‐19.^40^, ^41^, ^48^, ^80^ Babszky et al. reported that*Bacteroidetes spp*. in the feces has an anti‐inflammatory effect and possess protective features against severe COVID‐19 infection.^41^ Similarly, Dereschuk et al. reported that Less severe SARS‐CoV‐2 infection can be associated with the presence of *Bacillus subtilis spp*. in blood microbiotas.^48^ Also, Zuo et al. reported that*Faecalibacterium prausnitzii* has a negative correlation with the severity of the disease.

On the other hand, nine studies reported possible associations of some particular gut bacteria with more severe forms of COVID‐19.^42^, ^48^, ^50^, ^56^, ^66^, ^74^, ^80^, ^84^, ^85^ Dereschuk et al. reported that COVID‐19 infection was severe among patients with blood microbiota composition as follows:*E. coli, Bacillus, Campylobacter hominis, Pseudomonas, Thermoanaerobacter pseudethanolicus, Thermoanaerobacter iumthermosaccharolyticum*, and *Staphylococcus epidermis*.^48^ Also, loss of beneficial microorganisms was reported to increase potential pathogens for instance *Enterococcus*, especially among ICU patients.^50^ Moreira‐Rosário et al. reported a decrease in butyrate‐producing bacteria including;*Roseburia spp., Lachnospira spp*., and an increase in *Proteobacteria spp*. among moderate and severe COVID‐19 patients’ gut microbiota.^56^ Similarly, Reinold et al. found that a reduction in butyrate‐producing bacteria could be linked to more severe disease.^74^ Zhang et al. mentioned that the alterations in the gut microbiota of COVID‐19 patients can reduce the levels of l‐Isoleucine, SCFA (Short‐Chain Fatty Acid), and l‐Isoleucine even one month after recovery and this would result in more severe diseases.^85^ Finally, it was reported by Zuo et al. that*Coprobacilum spp., Clostridium Ramosum*, and *Clostridium hathewayi* were associated with more severe diseases.^80^

One similar systematic review stated that *Bifidobacterium, Bacteroides, Corynebacterium, Ruminococcus, Parabacteroides, Campylobacter, Clostridium, Ruminococcus, Rothia, Enterococcus, Megasphaera, Enterococcus*, and *Aspergillus* had high abundance among severe COVID‐19 patients while, *Lachnospira, Roseburia, Faecalibacterium, Eubacterium*, and *Firmicutes/Bacteroidetes* ratio had declined among severe COVID‐19 cases.^97^ Other similar studies also have noted the higher abundancy of opportunistic pathogens including;*Veilonella, Streptococcus, Rothia*, and *Actinomyces*,^80^, ^89^ and declining levels of beneficial commensal bacteria such as*Roseburia, Agathobacter, Fusicatenibacter*, and *Ruminococcaceae* among moderate to severe COVID‐19 patients.^80^

### 5.1 Associations between SARS‐CoV‐2 viral load and gut microbiota composition

Only two articles investigated the relations between gut microbiota and COVID‐19 viral load, one reported no relation between COVID‐19 viral load and GI microbioa,^40^ while the other one noted that in the gut microbiota, *Prevotellacopri*, and *Eubacterium dolichum* were associated positively with SARS‐CoV‐2 viral load, and *Streptococcus anginosus spp*., *Dialister spp., Alistipes spp., Ruminococcus spp., C. citroniae spp., Bifidobacterium spp., Haemophilus spp*., and *Haemophilusparainfluenza* were linked negatively to this load.^15^

### 5.2 Therapeutic probiotic implementation efficacy and safety in COVID‐19 patients

Thirteen studies included in our review assessed the effects of probiotic implementations on symptoms, morbidity, and mortality rates among COVID‐19 patients.^29^, ^33^, ^34^, ^35^, ^36^, ^37^, ^38^, ^39^, ^45^, ^70^, ^76^, ^77^, ^146^ Probiotics are live microorganisms whose administration in sufficient quantities has been demonstrated to ameliorate immune response, participate in metabolism, and balance the host microbiome.^147^, ^148^ Probiotics can be used as a complementary choice for the prevention and treatment of viral and bacterial infections.^149^ Many studies have reported that probiotics possess antiviral effects via a variety of mechanisms including; innate and adaptive immune system immunomodulation, mucosal protection maintenance, and pathogens inhibition through binding them.^150^ Among all probiotics mainly two genera of *Lactobacillus* and *Bifidobacterium* have been shown to be the two most common probiotics in use for the treatment of viral respiratory tract infections including; influenza virus, adenovirus, and respiratory syncytial virus.^151^, ^152^, ^153^

In our study, the most common probiotics used were *Lactobacillus* and *Bifidobacterium* as well and nine studies investigated the efficacy of these two genera among COVID‐19 patients.^29^, ^34^, ^35^, ^36^, ^38^, ^39^, ^45^, ^70^, ^76^ In addition, few studies had utilized other less common probiotics as follows; *Bos taurus*, *Morone, Leuconostoc, Lachesana, Limulus, Oryctolagus, Pentadiplandra, Rhamnosus*, and *Enterococcus*.^29^, ^38^, ^70^ Moreover, two studies utilized distinguished methods for balancing patients' altered microbiome including; Fecal microbiota transplantation (FMT)^33^ and washed microbiota transplantation (WMT),^37^ and two studies did not specify the exact type of studied probiotic.^77^, ^146^ Almost all these studies reported a diverse variety of probiotics' beneficial effects in combat against COVID‐19 symptoms, prognosis, and outcome.

Two studies reported that *Lactobacillus plantarum* metabolites have a high affinity for binding to ACE2 molecules, and *Lactobacillus plantarum* and *Lactococcus lactis* particles can bind with high affinity to SARS‐COV‐2 virus molecules thus they can be used against SARS‐CoV‐2 infection.^45^, ^70^ In one RCT using*Lactiplantibacillus plantarum*, and *Pediococcusacidilactici* strains, 53.1% of the probiotic‐receiving group achieved total remission while this number was significantly lower in the control group at 28.1%. In this study probiotic treatment was associated with reduced nasopharyngeal viral load, pulmonary infiltrations, and duration of symptoms, compared to the control group, also, probiotic treatment significantly increased anti‐SARS‐CoV‐2 IgM and IgG antibodies compared to the placebo group.^154^ In addition, taking*Lactobacillus rhamnosus GG* was mentioned to be protective against COVID‐19 and capable of reducing the severity of the disease.^36^ Another study reported that taking probiotic Lactobacillus and *Bifidobacterium* could produce organic acids, ethanol, and exopolysaccharides molecules that possess antiviral effects and may be useful in combating COVID‐19.^35^

Two studies reported the beneficial effects of *Bifidobacterium* in decreasing mortality rates and hospital admission duration of moderate/severe COVID‐19 patients, increasing blood antibody levels, and lowering inflammatory cytokines.^39^, ^76^ Similarly, one study reported that the use of probiotics was associated with a shorter duration of COVID‐19 illness and hospitalization and improved the conditions of COVID‐19 patients.^38^ A similar study assessed the effects of bacteriotherapy via the administration of *Streptococcus, Lactobacillus, and Bifidobacterium* strains. The authors reported that the risk of respiratory failure was 8 times lower in the bacteriotherapy group; additionally, the prevalence of ICU admissions and mortality rates were higher among the non‐bacteriotherapy patients.^119^ In addition, three studies noted the effectiveness of probiotics in treating diarrhea among COVID‐19 patients.^29^, ^34^, ^146^ Similar studies have reported consistent results with our study that probiotics can treat gut dysbiosis and thus mitigate the GI symptoms arising from it.^155^, ^156^ One RCT conducted in China reported that the use of *Bifidobacterium, Lactobacillus, Enterococcus*, and *Bacillus* tablets was associated with a better immune function and reduced secondary bacterial or fungal infection.^157^ Finally, FMT was reported to be a novel therapy with beneficial effects as follows; increasing microbial richness, restoring gut microbiota through decreasing *Proteobacteria*, and increasing *Bifidobacterium, Faecalibacterium*, and *Actinobacteria*, and alleviating GI symptoms.^33^ Similarly, WMT was reported to be effective and safe for COVID‐19 patients.^37^ Therefore, *Lactobacilli* and *Bifidobacteria* can be considered the main probiotics that can assist the most with balancing gut microbiome and possibly correct the dysbiosis caused by COVID‐19.

## 6 LIMITATIONS

This is an extensive systematic review of human Microbiota and COVID‐19 possible bidirectional associations. We screened a large number of available studies in several databases, evaluated their quality, and extracted their findings. However, our study has some limitations. First, we did not include non‐English articles, including Chinese studies in our review. Second, few included studies investigated, and took into account the comorbidities of COVID‐19 cases, as it has been shown that, comorbidities, and complications including; hypertension, cardiovascular diseases, hyperlipidemia, diabetes mellitus, and thromboembolic events can alter the gut, and lung microbiotas.^158^, ^159^ Third, only some studies had documented antibiotic use‐which most probably would have been high specifically during the first months of the pandemic‐ as they can also alter the human microbiome. Fourth, the possible causal association between the human microbiome and COVID‐19 was not certainly understood. Fifth, a variety of methods including; 16 S rRNA amplicon sequencing, qPCR, and waste water sampling had been used by the studies that can make it difficult to compare the bacterial alterations among the studies. Thus, further studies (e.g., longitudinal cohort studies) with larger sample populations, similar microbiome sampling methods are needed to investigate, and find the probable causative association between gut, and lung microbiota and COVID‐19. These studies can be conducted among both out‐patient, and inpatient COVID‐19 cases with mild to severe conditions, to enlighten this topic.

## 7 CONCLUSION

Our study shows that there was a significant difference in the composition of the URT, and gut microbiota in COVID‐19 patients compared to the general healthy population. In addition, specific microbiota compositions would be associated with COVID‐19 viral loads, and severity. These alterations‐which were mostly increasing patterns of opportunistic pathogens‐ can be further investigated to find possible causative associations between the human microbiome and COVID‐19, and used as a probable diagnostic and prognostic tools for COVID‐19 management. In addition, our study shows that probiotics use can be beneficial in terms of signs and symptoms management, and prognosis amelioration of COVID‐19 patients.

## AUTHOR CONTRIBUTIONS

**SeyedAhmad SeyedAlinaghi**: Conceptualization; writing – review and editing. **Arian Afzalian**: Writing – original draft. **Zahra Pashaei**: Writing – original draft. **Sanaz Varshochi**: Writing – original draft. **Amirali Karimi**: Writing – original draft. **Hengameh Mojdeganlou**: Writing – original draft. **Paniz Mojdeganlou**: Data curation. **Armin Razi**: Data curation; Resources. **Farzaneh Ghanadinezhad**: Data curation. **Alireza Shojaei**: Writing – original draft. **Ava Amiri**: Writing – original draft. **Mohsen Dashti**: Writing – original draft. **Afsaneh Ghasemzadeh**: Writing – original draft. **Omid Dadras**: Writing – review and editing. **Esmaeil Mehraeen**: Conceptualization; writing – review and editing. **Amir Masoud Afsahi**: Methodology.

## CONFLICT OF INTEREST STATEMENT

The authors declare no conflict of interest.

## TRANSPARENCY STATEMENT

The lead author Esmaeil Mehraeen affirms that this manuscript is an honest, accurate, and transparent account of the study being reported; that no important aspects of the study have been omitted; and that any discrepancies from the study as planned (and, if relevant, registered) have been explained.

## Supporting information

Supporting information.

## Data Availability

The authors stated that all information provided in this article could be shared. All authors have read and approved the final version of the manuscript [Esmaeil Mehraeen] had full access to all of the data in this study and takes complete responsibility for the integrity of the data and the accuracy of the data analysis. Esmaeil Mehraeen affirms that this manuscript is an honest, accurate, and transparent account of the study being reported; that no important aspects of the study have been omitted; and that any discrepancies from the study as planned (and, if relevant, registered) have been explained.
